# Deep Learning-Based Denoised MRI Images for Correlation Analysis between Lumbar Facet Joint and Lumbar Disc Herniation in Spine Surgery

**DOI:** 10.1155/2021/9687591

**Published:** 2021-07-29

**Authors:** Feng Gao, Mingcan Wu

**Affiliations:** ^1^Department of Spine Surgery, Tongji Hospital, Tongji University School of Medicine, Shanghai 200065, China; ^2^Spine Surgery, Yuyao People's Hospital of Zhejiang Province, Yuyao 315400, Zhejiang, China; ^3^Department of Radiology, Yuyao People's Hospital of Zhejiang Province, Yuyao 315400, Zhejiang, China

## Abstract

This work aimed to explore the relationship between spine surgery lumbar facet joint (LFJ) and lumbar disc herniation (LDH) via compressed sensing algorithm-based MRI images to analyze the clinical symptoms of patients with residual neurological symptoms after LDH. Under weighted BM3D denoising, Epigraph method was introduced to establish the novel CSMRI reconstruction algorithm (BEMRI). 127 patients with LDH were taken as the research objects. The BEMRI algorithm was compared with others regarding peak signal-to-noise ratio (PSNR) and structural similarity index (SSIM). Patients' bilateral LFJ angles were compared. The relationships between LFJ angles, lumbar disc degeneration, and LFJ degeneration were analyzed. It turned out that the PSNR and SSIM of BEMRI algorithm were evidently superior to those of other algorithms. The proportion of patients with grade IV degeneration was at most 31.76%. Lumbar disc grading was positively correlated with change grading of LFJ degeneration (*P* < 0.001). LFJ asymmetry was positively correlated with LFJ degeneration grade and LDH (*P* < 0.001). Incidence of residual neurological symptoms in patients aged 61–70 years was as high as 63.77%. The proportion of patients with severe urinary excretion disorders was 71.96%. Therefore, the BEMRI algorithm improved the quality of MRI images. Degeneration of LDH was positively correlated with degeneration of LFJ. Asymmetry of LFJ was notably positively correlated with the degeneration of LFJ and LDH. Patients aged 61–70 years had a high incidence of residual neurological symptoms after surgery, most of which were manifested as urinary excretion disorders.

## 1. Introduction

LDH is a common chronic spinal degenerative disease [1]. In recent years, the incidence of LDH has shown a significant upward trend, and a large number of studies have shown that LFJs are related to the occurrence of LDH [2]. In addition, studies have shown that the angle and asymmetry of LFJs are related to the occurrence of LDH [3]. Magnetic resonance imaging (MRI) technology is utilized in the diagnosis of LDH due to its noninvasiveness and multiple imaging angles. However, in the current research, there are generally cases where the results of imaging examinations do not match the patient's signs and symptoms. Moreover, due to the limited quality of MRI images, there are certain controversies about the occurrence of LFJ and LDH. Clinically, there are also cases where the images and physical signs do not match [4]. The quality of reconstructed images in traditional MRI algorithms is low. Some researchers applied compressed sensing (CS) theory to the reconstruction of MRI images and established the CSMRI algorithm, which can not only obtain the precise sparsity prior of the image but also capture the rich structural information of the image, and thus it is widely adopted in the field of MR image reconstruction. However, the CSMRI algorithm still cannot manage both image quality and calculation speed, and there is still room for further improvement in the quality of MR image reconstruction at low sampling rates [5].

At present, surgical methods are often adopted to treat LDH in clinic. Although surgical methods can significantly relieve the clinical symptoms of LDH patients, some patients still have residual neurological symptoms after surgery. The incidence of residual neurological symptoms after LDH is 5%–40%, with an average of 15%. The main manifestations are swelling, numbness, limp, and weakness of the lower limbs. Studies pointed out that the proportion of patients with lower extremity numbness after LDH operation was up to 21%–67%, and studies reported that patients with hip pain after LDH operation accounted for 63.1% [1]. At present, there are few studies on residual neurological symptoms in patients with LDH. Moreover, the proportion of symptoms after LDH is quite different, and further research on its symptoms is needed to provide a reference for the prognosis of LDH.

The deep ResNet method was introduced based on the deep learning algorithm to remove the Rician noise in MRI images and was applied to the diagnosis of LDH patients. From June 2018 to March 2020, 127 patients who underwent MRI diagnosis and were confirmed as LDH with residual neurological symptoms in our hospital's spine surgery were taken as the research objects. The relationship between LFJ, LDH, and residual neurological symptoms after surgery was explored to find out the cause of LDH and the residual neurological symptoms after surgery and provide a reference for the diagnosis and prognosis of LDH.

## 2. Materials and Methods

### 2.1. Research Objects

From June 2018 to March 2020, 127 patients who underwent MRI diagnosis and were confirmed as LDH with residual neurological symptoms in our hospital's spine surgery were taken as the research objects. 381 lumbar intervertebral discs and 381 pairs of LFJs and LFJs were measured.

The inclusion criteria in this study were defined as follows: patients diagnosed as LDH; patients without a history of lumbar spine surgery; patients who suffered from recurrent or persistent low back pain, sciatica, or its branch nerve compression symptoms 3 months after LDH surgery; and patients without prominent or nerve root compression or damage of original surgery segment after the surgery. The exclusion criteria could be determined as follows: patients whose MRI diagnosis images could not be found in the information query system of the hospital; patients with ankylosing spondylitis; patients with spinal tumors or lumbar tuberculosis; patients with failed LDH surgery; and patients accompanied by serious cardiovascular, cerebrovascular, liver and kidney, hematopoietic system or other serious diseases of other organs. The experimental process had been approved by the Ethics Committee of the hospital, and all subjects included in the study had signed the informed consent forms.

### 2.2. Denoising Algorithms for MRI Images Based on the Deep Learning

The traditional image denoising algorithms cannot completely remove the Rician noise in MRI images with relatively fuzzy image edge contours, and the deep learning mainly focuses on removing the Gaussian white noise. Therefore, the deep ResNet method was proposed based on the deep learning to remove the Rician noise in MRI images.

Gradient reduction could be found during the training of convolutional neural network (CNN) model, while the ResNet idea could solve this problem well. It was assumed that the input neural network of the ResNet was *x* and the function mapping was *H*(*x*); then the expression of the residual mapping *F*(*x*) was as follows:

(1) $$\begin{array}{c} F\left(x\right)=H\left(x\right)-x. \end{array}$$

The expression equation of the hidden layer could be written as follows:

(2) $$\begin{array}{c} H\left(x\right)=F\left(x\right)+x. \end{array}$$

It was expected to obtain the mapping *H*(*x*) by training the deep network, while the residual learning could fit the residual mapping *F*(*x*), and the residual learning equation was more suitable for solving the image denoising. The structure of ResNet is shown in Figure 1.

In the ResNet, the batch normalization (BN) method was used for intermediate preprocessing, so that the input of the previous layer was processed by BN before entering the next layer, which can avoid gradient explosion and improve the training speed. When the model was designed, BN was introduced after each convolutional layer. If one layer of the network was a d-dimensional input *x*={*x*_1_, *x*_2_,…, *x*_*d*_}, it could be normalized as in the following equation:

(3) $$\begin{array}{c} x_{k}=\frac{x_{k}-E\left(x_{k}\right)}{\sqrt{\text{Var}\left(x_{k}\right)}}, \end{array}$$

where *E*(*x*_*k*_) refers to the expectation and Var(*x*_*k*_) represents the variance.

Parameters *γ*_*k*_ and *β*_*K*_ were introduced to avoid influences on network learning features of this layer:

(4) $$\begin{array}{c} y_{k}=\gamma_{k}x_{k}+\beta_{k}. \end{array}$$

If BN was not introduced, the activation function layer *y* could be expressed as follows:

(5) $$\begin{array}{c} y=s\left(\omega x+b\right), \end{array}$$

where *w* refers to the weight; *b* and *s* represent the bias and activation function, respectively.

If the BN was introduced, the forward conduction could be written as in the following equation:

(6) $$\begin{array}{c} y=s\left(BN\left(\omega x+b\right)\right). \end{array}$$

The above equation could be normalized as follows:

(7) $$\begin{array}{c} y=s\left(BN\left(\omega x\right)\right). \end{array}$$

The gradient descent algorithm was the commonly used optimization algorithm in the neural network training process so as to obtain the minimum parameters of the loss function. The single-step weight and bias update expressions were as follows:

(8) $$\begin{array}{c} \omega_{k}⟶\omega_{k}^{\prime }=\omega_{k}-\left(\partial \frac{\delta C}{\delta \omega_{k}}\right),\\ b_{l}⟶b_{l}^{\prime }=b_{l}-\left(\partial \frac{\delta C}{\delta b_{l}}\right). \end{array}$$

The gradient descent algorithm was slow when the amount of data was large, so a stochastic gradient descent (SGD) algorithm was proposed. However, it adopted individuals to represent the overall change and cannot obtain the global optimal solution in each iteration. Therefore, the Adam algorithm was proposed in this study. The SGD algorithm updated all weights so that the learning rate remained stable during the network training. The Adam algorithm iteratively updated the weights of the neural network, which can solve the high-intensity noise or sparse gradient well.

As regards the Adam algorithm, the noise objective function was set to *f*(*θ*); the exponential moving average and square gradient were updated; and the deviation correction term was initialized.

(9) $$\begin{array}{c} v_{t}=\left(1-\beta_{2}\right)\sum_{i=1}^{t}\beta_{2}^{t-i}\cdot g_{i}^{2}, \end{array}$$

where *t* represents the time step; *β*_2_ refers to the exponential decay rate; and *g* represents the gradient.

After deviation correction, the expected value could be written as in the following equation:

(10) $$\begin{array}{c} E\left[v_{t}\right]=E\left[\left(1-\beta_{2}\right)\sum_{i=1}^{t}\beta_{2}^{i-1}\cdot g_{i}^{2}\right],\\ =E\left[g_{t}^{2}\right]\cdot \left(1-\beta_{2}\right)\sum_{i=1}^{t}\beta_{2}^{i-1}+\varsigma \\ =E\left[g_{t}^{2}\right]\cdot \left(1-\beta_{2}\right)+\varsigma . \end{array}$$

If the second moment *E*[*g*_*t*_^2^] was static, the *ς* value was 0.

The structure of the deep ResNet denoising model proposed in this study is shown in Figure 2. There were 15 network layers in total, 13 of which were hidden layers. Both the training image and the test image were grayscale ones. The size of the input layer was 3 × 3 × 1 × 64, including the activation function and the convolutional layer. The size of the hidden layer was 3 × 3 × 64 × 64, including activation function, BN, convolution, and pooling operations. The output layer size was 3 × 3 × 64 × 1, and the convolutional layer was reconstructed to output the image.

### 2.3. Degeneration Classification and Measurement Methods of LFJs and Lumbar Disc

The classification of LFJs could refer to the classification standards (0–3 levels) of LFJs degradation image defined by Song et al. [6]. L3/4, L4/5, and L5/S1 of the patients were scanned with MRI, and the scan line was parallel to the intervertebral space and passed through the corresponding LFJs. If the angle difference between two sides of LFJs of the same segment was greater than 7°, it was deemed that LFJs were asymmetric.

The grades of lumbar disc degeneration were divided into grades I–V [7]. The height of the first-level lumbar disc of the MRI image was to determine the degeneration grade. The vertical height of the center of the lumbar disc was calculated according to the two reference lines. According to the results of Brayda-Bruno et al. (2018) [8], the normal values of the height of each lumbar disc were 1.073 cm–1.247 cm for L3/4, 1.18 cm–1.272 cm for L4/5, and 0.939 cm–1.121 cm for L5/S1. It was determined as the slight decrease if the height was higher than 80% of the normal height. If the height was lower than 80% and higher than 60% of the normal height, it was deemed as a moderate decrease; and it was determined as gap collapse if the height was lower than 60% of the normal height.

### 2.4. Observation Indicators

The asymmetry of LFJs, LFJs degeneration grade, and lumbar disc degeneration were measured based on the MRI images of all patients. The basic clinical data, postoperative clinical manifestations, influencing factors, and nerve entrapment points were recorded for all patients.

### 2.5. Statistical Analysis

The experimental data was processed using SPSS 19.0 statistical software, the mean ± standard deviation ($\bar{x}$ ± *s*) was adopted to show the measurement data, and the *t*-test was employed for normal distribution. Spearman's rank correlation analysis was to analyze the lumbar disc degeneration grades, LFJs asymmetry, LFJs degeneration grades, LDH, and age, which did not obey the normal distribution (*α* = 0.005). The count data of patients with postoperative residual neurological symptoms of different ages and different genders were expressed in percentage (%), tested by the *χ*^2^ test. *P* < 0.05 indicated that the difference was considerable.

## 3. Results

### 3.1. Analysis of Denoising Performance of Different Algorithms

The proposed deep learning denoising algorithm was compared with the weighted stable matching (WSM) algorithm and denoising CNN (DnCNN) algorithm in terms of PSNR value (Figure 3(a)). The PSNR value of the image after denoising by the proposed algorithm was higher than those of the WSM algorithm and DnCNN algorithm under different noise intensities. Further analysis of the SSIM values of various algorithms (Figure 3(b)) revealed that the SSIM value of the image after denoising by the proposed algorithm was still higher than those of other algorithms. Based on the above results, it was obtained that the proposed algorithm had obvious advantages in denoising of the medical MRI images.

### 3.2. MRI Examination of Patients with Lumbar Disc Herniation

The MRI image of the LDH patient was compared with the MRI image of the normal human body, and the results are shown in Figure 4. The MRI image of the patient showed an obvious disc herniation and compression of the nerve root and the right dural sac.

### 3.3. The Correlation between the Grades of Lumbar Disc Degeneration and Lumbar Facet Joint

The proportion of patients in different lumbar disc degeneration grades was analyzed and compared, as shown in Figure 5. The proportion of patients with degeneration grade 4 was up to 31.76%. Further, there was an obviously positive correlation between the lumbar disc degeneration grade and the LFJ degeneration grade (*r* = 0.753, and *P* < 0.001).

### 3.4. Correlation between Lumbar Facet Joint Degeneration and Lumbar Disc Herniation

The correlation between LFJ degeneration grade and LDH was analyzed, and the results are shown in Table 1. They were extremely and negatively correlated (*r* = −0.306, and *P* < 0.001).

### 3.5. Correlation between Lumbar Facet Joint Asymmetry and Lumbar Disc Herniation

As shown in Table 2, LFJ asymmetry was extremely and positively correlated with the LDH (*r* = 0.543, and *P* < 0.001).

### 3.6. Distribution of Patients with Postoperative Residual Neurological Symptoms

A total of 81 patients with LDH had postoperative residual neurological symptoms, accounting for 63.77%. As age increased, the number of patients with postoperative residual neurological symptoms tended to increase and then decrease. Moreover, the patients aged 61–70 years accounted for the highest proportion (Figure 6). There were 18 male patients (22.22%) and 15 female patients (18.52%) with residual neurological symptoms in the age group of 61–70 years. In the entire age distribution, the proportion of males was higher than that of women, but the differences were not considerable (*P* > 0.05).

### 3.7. Symptoms of Postoperative Residual Neurological Symptoms

In this study, PRNSs of LDH were mainly manifested in waist pain, lower extremity radiating pain, buttock pain, waist movement limitation, lower extremity pain, lower extremity paresthesia, lower extremity weakness, severe urinary excretion disorder, and intermittent claudication (Figure 7). Most of patients suffered from serious urinary excretion disorders, reaching 71.96%.

## 4. Discussion

In this study, PSNR and SSIM values of the deep learning denoising algorithm were higher than those of other algorithms, showing that the quality of image treated with the deep learning denoising algorithm was higher [9, 10]. The proportion of patients with grade 4 degeneration was as high as 31.76%, and there was a dramatically positive correlation between the degeneration grade of lumbar disc and the degeneration grade of LFJ and age (*r* = 0.753, and *P* < 0.001). Ezemagu et al. [11] believed that herniation was caused when the pressure of the lumbar disc exceeded the load pressure. LFJs could protect the lumbar disc from damage due to excessive spine activity, so LFJ was positively correlated with herniation [12], which was similar to the results of this study. Cao et al. (2020) [13] found that the degeneration of LFJ could cause differences in the direction of the force on the lumbar disc nucleus pulposus, which could lead to different positions of LDH. There was a significantly positive correlation between LFJ degeneration grade and patient age (*r* = 0.694, and *P* < 0.001). There was a considerably negative correlation between LFJ degeneration and LDH (*r* = −0.306, and *P* < 0.001), and there was a significantly positive correlation between the asymmetry of LFJs and LDH (*r* = 0.543, and *P* < 0.001). The asymmetry of LFJs could cause the LFJs on one side to bear greater pressure, aggravate the degeneration and damage of the lumbar disc, and result in the occurrence of LDH [14]. LDH patients with PRNSs accounted for 63.77%, and patients aged 61–70 years accounted for the highest proportion, which was consistent with the results of Wu et al. (2020) [15]. The proportion of patients with severe urinary excretion disorders accounted for more than 71.96%, which might be because most of patients were 61–70 years old and some older patients suffered from different degrees of prostate disease.

## 5. Conclusion

The deep ResNet method was introduced based on the deep learning algorithm to construct a deep learning denoising algorithm for MRI image. The constructed denoising algorithm was applied to the diagnosis of LDH patients. The correlations among LFJ angle, lumbar disc degeneration, and LFJ degeneration were analyzed. However, there were still some shortcomings in this study. The age span of the observation objects was large, and the different age groups were not classified and analyzed with the grading of intervertebral disc degeneration and the degree of degeneration of LFJs. It will supplement related data in the future research. In summary, the deep learning denoising algorithm can improve the quality of MRI image. The degeneration of the lumbar disc was extremely and positively correlated with the degeneration of LFJ; the asymmetry of LFJs was significantly and positively correlated with LFJ degeneration grade and LDH; and PRNSs were mainly concentrated in the people aged 61–70 years. This work provides a reference basis for the diagnosis, treatment, and prognosis of LDH [16–18].

## Figures and Tables

**Figure 1:** The structure of residual network.

**Figure 2:** The structure of the deep ResNet denoising model.

**Figure 3:** Comparison of PSNR and SSIM values under different algorithms. *Note.* (a) illustrates the comparison results of PSNR, and (b) discloses the comparison results of SSIM.

**Figure 4:** MRI of patients with LDH. (a) shows an MRI image of lumbar disc of a normal human body; (b) shows an MRI image of a male patient aged 42 years with L4/5 disc herniation; (c) shows an MRI image of L3/4 disc herniation for a female patient aged 39 years; and (d) shows an MRI image of L5/S1 right disc herniation for a male patient aged 64 years.

**Figure 5:** Distribution of lumbar disc degeneration grade and its correlation with LFJ degeneration grade. (a) illustrates the analysis of the proportion of patients in different grades of lumbar intervertebral disc degeneration; and (b) illustrates the correlation between the grades of lumbar intervertebral disc degeneration and LFJ degeneration.

**Figure 6:** Analysis of the age and gender distribution of patients with postoperative residual neurological symptoms.

**Figure 7:** Symptoms of postoperative residual neurological symptoms. Note: A, B, C, D, E, F, G, H, and I in the horizontal coordinate refer to waist pain, hip pain, lower extremity radiating pain, lower extremity pain, waist movement limitation, lower extremity weakness, lower extremity paresthesia, intermittent claudication, and severe urinary excretion disorder, respectively.

**Table 1:** Correlation between LFJ degeneration and LDH.

LFJ degeneration grade	LDH		
	LDH (52 cases)	Lumbar disc bulging (69 cases)	No obvious herniation or bulging (6 cases)
Grade 0	14 (26.92%)	20 (38.46%)	2 (3.85%)
Grade 1	21 (40.38%)	31 (59.62%)	4 (7.69%)
Grade 2	10 (19.23%)	11 (21.15%)	0 (0)
Grade 3	7 (13.46%)	7 (13.46%)	0 (0)

**Table 2:** Correlation between LFJ asymmetry and LDH.

LFJs asymmetry	LDH		
	LDH (52 cases)	Lumbar disc bulging (69 cases)	No obvious herniation or bulging (6 cases)
L3/4	25 (48.08%)	23 (44.23%)	2 (3.85%)
L4/5	9 (17.31%)	15 (28.85%)	3 (5.77%)
L5/S1	18 (34.62%)	31 (59.62%)	1 (1.92%)

## Data Availability

The data used to support the findings of this study are available from the corresponding author upon request.
